The article "Influence of Health Education Based on IMB on Prognosis and Self-Management Behavior of Patients with Chronic Heart Failure" was retracted in 2023. Reasons: unreliable results or conclusions; lack of ethics approval or compliance; concerns about the data; concerns about the peer review.

# Influence of Health Education Based on IMB on Prognosis and Self-Management Behavior of Patients with Chronic Heart Failure

**DOI:** 10.1155/2022/8517802

**Published:** 2022-04-08

**Authors:** Wei Liu, Yan Zhang, Hai-jing Liu, Tian Song, Song Wang

**Affiliations:** ^1^Nursing Department, Qiqihar Medical University, Qiqihar, 161006 Heilongjiang, China; ^2^Cardiovascular Internal Medicine Ward 6, The Second Affiliated Hospital of Qiqihar Medical University, Qiqihar, 161006 Heilongjiang, China; ^3^Emergency Medicine, The Third Affiliated Hospital of Qiqihar Medical University, Qiqihar, 161006 Heilongjiang, China; ^4^Internal Medicine Ward 5, Staff Hospital of Qiqihar Machine Tool Group Co. Ltd., Qiqihar, 161006 Heilongjiang, China

## Abstract

As the contemporary society is increasingly entering an aging society, heart failure, as a common disease in the elderly population, has an increasing impact on people. The common one is mainly chronic heart failure. Coupled with the influence of various complications, such as hypostatic pneumonia and venous thrombosis, the mortality and hospital admission rates of patients are very high. Moreover, the current technology is not very effective for the prevention and treatment of chronic heart failure. The per capita consumption level of ordinary people in China is low, and it is not suitable to promote high-cost treatment programs. Based on this, this paper proposes the intervention management of mental failure patients under the intervention of health education based on IMB, in order to explore the impact of the intervention of health education on patients. The research in this paper selected 112 patients with chronic heart failure who were admitted to the cardiovascular ward of a city public hospital in 2017 and divided the patients into two groups. One group received health education intervention, which was the intervention group. The other group was the control group. The control group was given routine education and nursing. The experimental results of this paper show that the satisfaction of the intervention group is higher, accounting for 85.3%, and the satisfaction of the control group is lower than that of the intervention group, about 67.9%. Dissatisfaction with health education and the probability of short-term readmission were higher than those in the intervention group.

## 1. Introduction

Chronic heart failure is a common clinical circulatory system disease, which mostly occurs in middle-aged and older. It is usually the long-term abnormal function of the heart that reduces the ability of the heart muscle to contract and causes poor blood circulation. Most patients had other types of cardiovascular disease, as heart failure was often caused by exacerbations of other cardiovascular diseases and was the leading cause of death in patients. A large number of studies at home and abroad show that chronic heart failure has become a global public health problem. Chronic heart failure patients have the characteristics of repeated attacks, long course of disease, lack of effective treatment, complex pathogenesis, and many pathogenic factors. The development of the disease can lead to a series of complications, affecting a person's survival, seriously affecting family life, and creating a double burden. It is a severe clinical syndrome with poor recovery prospects and high rates of unplanned readmissions and deaths. In recent years, in addition to significant progress in the research and development of targeted drugs, no effective treatment for chronic heart failure has been found in terms of clinical symptoms. Overseas studies have shown that more than 27% of patients with chronic heart failure return to the hospital within 3 to 6 months. The five-year survival rate for clinically diagnosed patients is only about 50%. In severe cases, the one-year mortality rate is as high as 50%. Therefore, treatment of chronic heart failure should not be limited to symptom relief, but should focus on multiple aspects of a patient's life to reduce mortality and readmission rates. Today, the medical model has entered the stage of biopsychosocial medicine. In the era of biopsychosocial medicine, health education plays an important role in the hospital system. Health education is based on the service center of medical institutions and takes people as the guiding ideology. Through daily education and communication, patients are introduced to the concept of health in a planned and purposeful manner. The goal is to change unhealthy behaviors in patients and improve their quality of life and well-being [1]. Appropriately intervene in patients' daily behavior through health education, change their concept, and thus, change their daily behavior. It can effectively improve the patient's self-care ability, reduce pain, relieve symptoms such as psychological depression, improve the quality of life of the patient, and indirectly reduce the cost of treatment.

The article "Influence of Health Education Based on IMB on Prognosis and Self-Management Behavior of Patients with Chronic Heart Failure" was retracted in 2023. Reasons: unreliable results or conclusions; lack of ethics approval or compliance; concerns about the data; concerns about the peer review.

The IMB model mainly affects the patient's self-management behavior through three elements: information, motivation, and behavioral ability. Information is a prerequisite for healthy behavior. In this study, we used three scales to identify subjects' common weaknesses in disease knowledge, daily life style, and related skills. And it adopts the method of issuing health education manuals to respond to the subjects' confusion and misunderstanding of relevant knowledge in a timely manner. Through individual guidance, let them establish correct understanding, change misconceptions, and fully understand the occurrence and development of diseases. It helps patients reduce psychological stress and pain. It can provide an effective approach to health education to improve the lives of patients with chronic heart failure.

In this study, the benefits of a doctor-nurse collaborative health education model were fully exploited. The traditional method of health education only carried out by nurses has been replaced by the method of cooperation between doctors and nurses, deepening and broadening health education from different angles and achieving better results in health education. Based on the IMB model, we can solve the confusion and misunderstanding of patients in various ways, establish a correct understanding, and reduce psychological pressure.

## 2. Related Work

As the current society begins to enter the aging process, heart failure, which is multiple and accompanied by other diseases, has become one of the key points of the world's attention. Scholars at home and abroad have carried out in-depth research on it. Among them, Zhang et al. evaluated the effect of conductive health education on the self-management behavior of elderly patients with hypertension and gastric ulcer. The results show that conductive health education can effectively improve the self-management behavior of elderly patients with hypertension and gastric ulcer [2]. Paying attention to the self-care skills of patients with chronic diseases, especially those with cardiovascular diseases, based on educational interventions will help them improve their conditions. The Barkhordari-Sharifabad study investigated the effects of promoting health literacy through virtual education on self-care behaviors in patients with heart failure. The intervention included four themes on self-care issues in text, photos, animations, and short films. Participants will be provided with a topic link each week. After the link is sent, through the cyberspace system, the necessary follow-up on the acquisition and understanding of the information and its application is carried out, and the correct self-care essentials results are emphasized. According to the paired *t*-test results, the mean scores of overall self-care in both groups increased after the intervention compared to before the intervention (*P* < 0.05) [3]. The safety and efficacy of aerobic exercise in heart failure (HF) patients with atrial fibrillation (AF) have not been well evaluated. Luo et al.'s study investigated whether the outcomes of high-frequency training differed by atrial fibrillation. In the overall population, there were no significant differences in the incidence of AF by randomization to treatment assignment or baseline AF status (all *P* > 0.10). There was no interaction between atrial fibrillation and exercise training on functional status or clinical outcome measures (all *P* > 0.10). Atrial fibrillation in patients with chronic HF was associated with older age, lower exercise capacity at baseline, and a higher overall frequency of clinical events, but did not respond differently to training-induced changes in clinical outcomes or exercise capacity [4]. The cost-effectiveness of heart failure management interventions can be further understood by combining the expected benefits and costs of future survival. The Maru et al.'s study compared long-term costs (mean intervention duration = 12 months) per quality-adjusted life-year (QALY) obtained from home (HBI) and specialist clinic intervention (CBI) in elderly patients discharged with heart failure (mean age = 71 years). Compared with CBI (outpatient specialist HF clinic-based intervention), HBI (mostly home-based, but not exclusively home-based) has a potential long-term cost-effectiveness threshold of A$50,000/QALY in elderly heart failure patients willing to pay [5]. A novel biomarker, human epididymal protein 4 (HE4), shows prognostic value in patients with acute heart failure (HF). Piek et al. measured HE4 levels in patients with chronic heart failure (CHF) and correlated it with HF severity, renal function, and biomarkers of HF to determine its predictive value [6]. Nymo et al. seek to use a systematic approach to assess whether a panel of biomarkers can improve outcomes in patients with heart failure (HF) and ischemic reduced ejection fraction, as required by recommendations for validation of new biomarkers. In conclusions, in the specific HF patient population studied, a multimarker approach using a specific biomarker panel measured has limited clinical value in determining the risk of adverse future outcomes [7]. The studies of the scholars all have the corresponding advantages of improving the diagnosis and treatment of patients with heart failure, but the research is time-consuming, and the experimental data are limited, which cannot represent the whole, and suitable and sufficient samples are not easy to gather.

The article "Influence of Health Education Based on IMB on Prognosis and Self-Management Behavior of Patients with Chronic Heart Failure" was retracted in 2023. Reasons: unreliable results or conclusions; lack of ethics approval or compliance; concerns about the data; concerns about the peer review.

## 3. Detection of Chronic Heart Failure

### 3.1. Preprocessing of Medical Images Based on Chronic Heart Failure

Medical images are mostly used for medical treatment or medical research. The purpose of medical image processing is to restore images with insufficient clarity, to highlight some feature information, or to classify images, etc.

#### 3.1.1. Image Filtering

In the process of image formation or transmission, the image will be affected by various factors, resulting in poor quality [8]. Therefore, smoothing filtering is used to remove part of the noise [9]. Smoothing filtering is mainly achieved by smoothing out high-frequency details in the image to reduce contrast and enhance the details of low-frequency parts. Use *G*(*x*, *y*) to represent the filter, *L*(*x*, *y*) to represent the input image sample, and the expression of the output image *T*(*x*, *y*) at this time is:

(1) $$\begin{array}{c} T\left(x,y\right)=G\left(x,y\right)\cdot L\left(x,y\right)=\overset{i-1}{\underset{r=1}{\sum }}\overset{j-1}{\underset{s=0}{\sum }}G\left(r,s\right)*L\left(x-r.y-s\right). \end{array}$$

Among them, *G*(*x*, *y*) can select appropriate filters through different selection requirements, such as median or mean filter.

Median filtering is a signal processing method that, in some cases, overcomes the nonlinear problem of blurring image details caused by the previous filter. The specific implementation of median filtering is relatively simple because it reduces the dependence on the statistical properties of the image [10–12]. In contrast, median filtering mainly refers to the method of replacing the gray value of the central pixel with the median value [13]. As can be seen in Figure 1, median filtering is implemented with a sorting method for pixel gray levels in a sliding window [14].

Using *A*1, *A*2, ⋯, *Ai* to represent the domain gray value of a point (*A*, *B*), the formula of median filtering is expressed as follows:

(2) $$\begin{array}{c} G\left(A,B\right)=\text{Med}\left[A1,A2,\cdots ,Ai\right]. \end{array}$$

Median filtering has advantages in reducing noise and preserving signal compared to mean and Gaussian filtering. Therefore, by choosing median filtering for image filtering, isolated points can be eliminated.

After smoothing and denoising the image using filtering techniques, image enhancement techniques in the zero domain or frequency domain can also be used to highlight the contrast between the object and the background and to emphasize the information describing the strong features of the image [15–17].

#### 3.1.2. Image Interpolation

When analyzing medical images, it is necessary to view a specific angle, or the area to be viewed may actually be just a section of the image. This requires the use of grayscale interpolation techniques to construct a viewing plane based on predictions of new data points from known data points [18–20]. Image comparison analysis in medical image classification requires the use of interpolation techniques, also known as resampling or resampling [21]. There are three common modes of grayscale interpolation of two-dimensional images, nearest neighbor interpolation, bilinear interpolation, and cubic polynomial interpolation. The principle of grayscale interpolation of two-dimensional images is shown in Figure 2.

The article "Influence of Health Education Based on IMB on Prognosis and Self-Management Behavior of Patients with Chronic Heart Failure" was retracted in 2023. Reasons: unreliable results or conclusions; lack of ethics approval or compliance; concerns about the data; concerns about the peer review.

### 3.2. Shape Feature Extraction of Medical Images

There are two main approaches to describe shape features: boundary-based and region-based [22]. Boundary-based methods use only the outer edges of the shape, while region-based methods use the entire area of the shape.

#### 3.2.1. Boundary-Based Shape Features

The boundary of the image can be reflected by the discontinuity of grayscale. The CT image is a grayscale image. If a pixel is a boundary point, the value of its gradient vector is generally outside a certain range [23]. After decades of development, many experts and scientists have proposed edge detection operators to find edge points and describe edge features [24]. Two classical principles for finding edge points are widely used: one is the first derivative of the maxima of the derivative, and the other is that the second derivative of the point is zero [25].

*(1) Edge Detection Operator with First-Order Differential*. The boundary is extracted by calculating the gradient of each pixel in the image corresponding to the maximum value of the first-order differential [26]. The commonly used first-order differential detection operators include Robert and Sobel operators.

The Robert operator locates the edge by the local difference operator. The formula for the Robert operator is:

(3) $$\begin{array}{c} J\left(y\left(A,B\right)\right)={\left|{\left[y\left(A,B\right)-y\left(A+1,B+1\right)\right]}^{2}+{\left[y\left(A+1,B\right)-y\left(A,B+1\right)\right]}^{2}\right|}^{1/2}. \end{array}$$

The calculated value of *J*(*y*(*A*, *B*)) can detect the point at the edge, and its size reflects the local change of the image.

Another commonly used first-order differential operator is the Sobel operator, which detects edges by computing neighborhood differences [27]. The weighting method is generally used in the calculation. Weighting the influence of the position of the pixels can reduce the degree of edge blur, so the effect is better. If the weights are different, the results of the operators will be different [28, 29]. The size of the weights is related to different distances, and small distances have a large impact on the neighborhood and the current pixel [30–33]. In the calculation, the difference value is obtained by calculating the average value of the gray level of the pixel by weighting, and the expression is:

(4) $$\begin{array}{c} Q=\sqrt{Q_{A}^{2}+Q_{B}^{2}}, \end{array}$$

(5) $$\begin{array}{c} Q_{A}=\left[y\left(A-1,B-1\right)+2y\left(A,B-1\right)+y\left(A+1,B-1\right)\right], \end{array}$$

(6) $$\begin{array}{c} Q_{B}=\left[y\left(A+1,B-1\right)+2y\left(A+1,B\right)+y\left(A+1,B+1\right)\right]. \end{array}$$

In the formula, *A* and *B* represent two directions, and analyzing their directions can reveal the extended edge information needed to select two spaced rows or columns for difference calculation.

*(2) Second-Order Differential Detection Operator*. Laplacian is a common direction-independent second-order differential detection operator, which is mainly used for 3 × 3 convolution of edge extraction. It is a direction-independent edge detection operator developed by selecting thresholds and finding boundary points based on the principle of zero-crossing of second-order differential derivatives [34]. Let *y*(*A*, *B*) represent the image and *T*(*A*, *B*) represent the Laplacian edge operator, and its expression formula is:

(7) $$\begin{array}{c} T\left(A,B\right)=y\left(A-1,B\right)+y\left(A+1,B\right)+y\left(A,B-1\right)+y\left(A,B+1\right)-4y\left(A,B\right). \end{array}$$

In the formula, to get edge information, it is only necessary to take the opposite sign of adjacent pixels. And *y*(*A*, *B* + 1) represents the filtered image of *y*(*A*, *B*).

*(3) Optimization Detection Operator*. Compared with the first-order and second-order difference detection operators, the Canny operator is a multistage optimization operator. It measures the product of signal-to-noise ratio and localization, but since it can achieve filtering, enhancement, and detection at the same time, the actual computation is cumbersome [35]. However, the Canny operator can only detect the edge in the image once, and it will also mark the possible image noise as the edge. The specific implementation steps are as follows.

The article "Influence of Health Education Based on IMB on Prognosis and Self-Management Behavior of Patients with Chronic Heart Failure" was retracted in 2023. Reasons: unreliable results or conclusions; lack of ethics approval or compliance; concerns about the data; concerns about the peer review.

First, to define a one-dimensional Gaussian filter function *g*(*A*), through which the image is smoothed:

(8) $$\begin{array}{c} g\left(A\right)=\frac{1}{\sqrt{2\pi \alpha }}ex\left(-\frac{A^{2}}{2\alpha^{2}}\right). \end{array}$$

Secondly, it is assumed that the convolution templates of the first-order difference are *W*1 and *W*2, according to which the corresponding gradient direction and amplitude can be calculated. It is required to take the point with the largest local gradient, which needs to be obtained by suppressing the amplitude, which can better preserve the refined edge.

$W1=\left|\begin{array}{cc} -1, & -1\\ 1, & 1 \end{array}\right|$ and $W2=\left|\begin{array}{cc} 1, & -1\\ 1, & -1 \end{array}\right|$, and their corresponding directions and magnitudes are:

(9) $$\begin{array}{c} F1\left(i,j\right)=y\left(i,j\right)\cdot W1\left(A,B\right), \end{array}$$

(10) $$\begin{array}{c} F2\left(i,j\right)=y\left(i,j\right)\cdot W2\left(A,B\right), \end{array}$$

(11) $$\begin{array}{c} \beta \left(i,j\right)=\sqrt{F_{1}^{2}\left(i,j\right)+F_{2}^{2}\left(i,j\right)}, \end{array}$$

(12) $$\begin{array}{c} \chi \beta =\text{arc}\left[\frac{F2\left(i,j\right)}{F_{1}\left(i,j\right)}\right]. \end{array}$$

Finally, edges are detected by thresholding.

#### 3.2.2. Regional Shape Features

The region-based shape description is mainly described by extracting the features of the region of interest. Commonly used extraction methods include roundness, moment of inertia, and geometric moment features.

*(1) Roundness [36]*. Assuming that the area of a circle is *P* and the perimeter is *S*, the perimeter will change with the change of the outside world. In the case of the same area, the perimeter is the shortest, and the shape features can be expressed most densely at this time. The definition formula of roundness, that is, the density *E*, is:

(13) $$\begin{array}{c} E=\frac{S^{2}}{\left(4\pi P\right)}. \end{array}$$

*(2) Moment of Inertia [37]*. In terms of physical definition, the concept based on the center of gravity can represent the center of mass (*ZA*, *ZB*) of the center of gravity of the grayscale image *y*(*A*, *B*), and the expression is as follows:

(14) $$\begin{array}{c} ZA=\frac{\sum_{A=1}^{i}\sum_{B=1}^{j}A\cdot y\left(A,B\right)}{\sum_{A=1}^{i}\sum_{B=1}^{j}y\left(A,B\right)}, \end{array}$$

(15) $$\begin{array}{c} ZB=\frac{\sum_{A=1}^{i}\sum_{B=1}^{j}B\cdot y\left(A,B\right)}{\sum_{A=1}^{i}\sum_{B=1}^{j}y\left(A,B\right)}. \end{array}$$

Assuming that the moment of inertia around the center of mass (*ZA*, *ZB*) is *L*(*ZA*, *ZB*), the definition formula is as follows:

(16) $$\begin{array}{c} L\left(ZA,ZB\right)=\overset{i}{\underset{A=1}{\sum }}\overset{j}{\underset{B=1}{\sum }}{\left[\left(A,B\right)-\left(ZA,ZB\right)\right]}^{2}y\left(A,B\right), \end{array}$$

(17) $$\begin{array}{c} L\left(ZA,ZB\right)=\overset{i}{\underset{A=1}{\sum }}\overset{j}{\underset{B=1}{\sum }}\left({\left(A-ZA\right)}^{2}+{\left(B-ZB\right)}^{2}\right)Y\left(A,B\right). \end{array}$$

The formula of moment of inertia is normalized, and the moment of inertia is expressed as *NM* as follows:

(18) $$\begin{array}{c} NM=\frac{\sqrt{L\left(ZA,ZB\right)}}{w}, \end{array}$$

(19) $$\begin{array}{c} NM=\frac{\sqrt{\sum_{A=1}^{i}\sum_{B=1}^{j}\left({\left(A-ZA\right)}^{2}+{\left(B-ZB\right)}^{2}\right.y\left(A,B\right)}}{\sum_{A=1}^{i}\sum_{B=1}^{j}y\left(A,B\right)}. \end{array}$$

In the formula, *w* = ∑_*A*=1_^*i*^∑_*B*=1_^*j*^*y*(*A*, *B*) is the quality of the image, which can represent the sum of all grayscale values of the image.

*(3) Geometric Moment [38]*. Suppose *y*(*A*, *B*) is a piecewise continuous probability density distribution function, and (*i* + *j*) represents a two-dimensional continuous random function. The unique moment sequence w*ij* of each order of the function can be determined by the density distribution function. Therefore, the definition formula of the origin moment w*ij* of (*i* + *j*) is:

(20) $$\begin{array}{c} Wij=\int \int A^{i}B^{j}y\left(A,B\right)rArB. \end{array}$$

The central moment is:

(21) $$\begin{array}{c} Vij=\int \int {\left(A-\bar{A}\right)}^{i}{\left(B-\bar{B}\right)}^{j}y\left(A,B\right)rArB. \end{array}$$

In Formula (21), $\bar{A}=w10/w00$, $\bar{B}=w01/w00$, and $\left(\bar{A},\bar{B}\right)$ represent the centroid of the image *y*(*A*, *B*).

The article "Influence of Health Education Based on IMB on Prognosis and Self-Management Behavior of Patients with Chronic Heart Failure" was retracted in 2023. Reasons: unreliable results or conclusions; lack of ethics approval or compliance; concerns about the data; concerns about the peer review.

Normalize the central moment:

(22) $$\begin{array}{c} \begin{array}{c} \delta \text{ij}=Vij/V00,\\ k=i+j+2/2,i+j=2,3,.\cdots \end{array} \end{array}$$

### 3.3. Basic Flow of Medical Image Processing

The main modules of feature extraction and classification of medical images are image preprocessing, feature extraction, and classification. Its algorithm also focuses on feature extraction and classification. The main steps in extracting features from medical images are as follows.

1. Extract the features of the processed medical image, select appropriate feature information, and form a feature vector
2. According to the feature information to be classified, a category model is established between the images
3. Develop classification algorithms, and develop classifiers through similarity measures, neural networks, support vector machines, and other methods
4. Train the classifier by inputting the image data to be classified, called training images and test images, respectively
5. The classification result of the output image

The main process of classifying medical images is shown in Figure 3.

### 3.4. The Theoretical Basis of IBM

The IMB model recognizes that there are three main factors that are important in the initiation and maintenance of healthy behaviors: accurate information, personal and social motivation (including attitudes, intentions, and norms), and behavioral skills. This is shown in Figure 4.

Informational factors are a prerequisite in the behavior change process, including events, inspirations, or theories related to the behavior change process. However, in practice, it was found that the interaction between information and behavioral change was not significant when individuals had good knowledge. This theoretical model suggests that information and behavioral change are affected by skill complexity and that behavioral change does not have to be information-based, but when complex behavioral skills are required, information must be involved in an individual's behavioral change.

The article "Influence of Health Education Based on IMB on Prognosis and Self-Management Behavior of Patients with Chronic Heart Failure" was retracted in 2023. Reasons: unreliable results or conclusions; lack of ethics approval or compliance; concerns about the data; concerns about the peer review.

Motivational factors include personal and social motivations. Personal motivation refers to the subject's forward-looking perception of behavior change, including his attitude, willingness to change, and perception of its importance, whereas social motivation includes support from family, friends, and relatives and their perception of behavioural change; in other words, the attitudes and opinions of people outside the subject. This theoretical model suggests that only when individuals possess high levels of information and related behavioral skills should they be strongly motivated to prevent behavioral change and maintain it.

The IMB model argues that behavioral change is a continuous process where each factor is intertwined. That is, an individual acquires the appropriate level of accurate knowledge, has a positive attitude and motivation, changes behavior with the support of family members, and acquires relevant skills.

This intervention was used in this study not only because it is widely used abroad but also because it accounts for the variability in the causes of behavioral change and the interaction between various factors.

## 4. Experiment of IMB-Based Health Education on Patients with Chronic Heart Failure

### 4.1. Improved Research Framework Based on the Original IMB

This intervention is based on the three phases of the IMB model: information transfer, motivation building, and skills transfer. The aim was to understand the impact of the IMB model on risk perception, medical coping, and self-management in patients with chronic heart failure. The flow of IBM's intervention structure is shown in Figure 5.

### 4.2. Health Education Based on IMB

#### 4.2.1. Determination of the Study Population

The number of heart failure patients admitted to a public hospital in a city within one year was taken as the research object of this work. Patients who met the inclusion criteria were selected from the Department of Cardiology.

1. Inclusion criteria

First, it meets the diagnostic criteria for heart failure.

The second is a person with a cardiac function class II to IV.

Third, people who are ≥18 years old, are conscious, can speak fluently, and can communicate by telephone.

Fourth, primary school or above.

Fifth, the course of disease ≥3 months.

Sixth, participate voluntarily and sign the informed consent.

(2) Exclusion criteria

First: people with cognitive impairment or mental illness.

Second: people with other serious systemic diseases, such as lung disease and malignant tumors.

The article "Influence of Health Education Based on IMB on Prognosis and Self-Management Behavior of Patients with Chronic Heart Failure" was retracted in 2023. Reasons: unreliable results or conclusions; lack of ethics approval or compliance; concerns about the data; concerns about the peer review.

Third: people with heart failure due to alcoholism or systemic diseases.

Fourth: people with severe hearing or visual impairment.

Fifth: people who live in nursing homes for a long time.

#### 4.2.2. Confirmation of the Number of Samples

(23) $$\begin{array}{c} I1=I2=2{\left[\frac{\left(V\varepsilon +V\gamma \right)}{\varphi /\phi }\right]}^{2}+\frac{1}{4}V\varepsilon^{2}. \end{array}$$

Among them, *I* is the content of the sample, *φ* is the mean difference between the two samples, and *ϕ* is the standard deviation of the population.

#### 4.2.3. Research Group

Control group (usual care and health education): patients received routine care and health education in cardiology during their hospital stay. It includes medication care, dietary care, symptomatic care during hospitalization, and discharge guidance. Patients receive a “Heart Failure Health Education Handbook” that contains information on medication management and self-efficacy.

Intervention group (on the basis of routine health education, implement health education in the mode of cooperation between doctors and nurses): the attending physician and the attending nurse jointly implement health education for the patients. The physician and the nurse should not only divide the labor but also cooperate, communicate with each other, learn from each other, and establish a cooperation model between the physician and the nurse. Leadership of the team rests with the senior nurse. In order to ensure the fairness and impartiality of the two health education methods, the training plan was jointly formulated by the department head and senior nurses, and the training and assessment of the health education knowledge of chronic heart failure were jointly carried out by the nurses in charge and senior doctors. The ward environment, medical equipment, treatment, nursing, and rules and regulations are the same, and the staff levels of the two wards are also the same, which ensures that the two groups of patients participate in health education with the same propaganda content in different ways.

### 4.3. Intervention Methods for Heart Failure Patients and the Basic Situation of the Samples

The research data were processed and analyzed with SPSS17.0 statistical software. Quantitative data are expressed as mean ± standard deviation, and *t*-test was used to compare the observed indicators between the two groups; qualitative data were analyzed as percentages. Differences were considered statistically significant at *P* < 0.05.

According to the basic conditions of the two groups of patients in Table 1, the general information of the two groups of patients was collected. It includes the average age, gender, educational level, occupation, family monthly income, and reimbursement method of hospitalization expenses of the two groups of chronic heart failure patients. The gender comparison of the two groups of patients is relatively average. The educational background of the patients is mostly below the primary school level, the income range is 2000-4000, and the occupation is mostly concentrated in farmers. There was no significant difference between the two groups of patients (*P* > 0.05), which was comparable.

The article "Influence of Health Education Based on IMB on Prognosis and Self-Management Behavior of Patients with Chronic Heart Failure" was retracted in 2023. Reasons: unreliable results or conclusions; lack of ethics approval or compliance; concerns about the data; concerns about the peer review.

From the comparison probability map of disease data in Figure 6, we have a preliminary understanding of the basic conditions of the two groups of patients. From the overall comparison of cardiac function classification, years of illness, and the number of comorbidities, the difference between the two groups is not large, but there are individual differences. This may affect the bias of later experimental data. Second, most of the patients' disease years were concentrated in 1 to 3 years, and most of the patients who participated in the experiment had 2 to 3 combined diseases.

## 5. Experimental Analysis of IMB-Based Health Education on Patients with Chronic Heart Failure

### 5.1. Emotional Comparison of Two Groups of Chronic Heart Failure Patients Based on IMB Health Education

Table 2 and Table 3 are the negative emotion comparison data of the two groups of patients at the time of admission and discharge. In the control group, the anxiety score was 3.1 ± 0.4 and the negative emotion score was 3 ± 0.5 at admission. The anxiety score of the patients in the intervention group was 3 ± 0.5, and the negative emotion score was 2.9 ± 0.4 at admission. After the two groups received treatment and were discharged from hospital for a period of time, the quality of life questionnaire was conducted again. The anxiety score of the control group was 2 ± 0.5, and the negative emotion score was 2 ± 0.4. The anxiety score of the experimental group was 1.8 ± 0.5, and the negative emotion score was 1.7 ± 0.5, and the difference was statistically significant *P* < 0.05. Anxiety and negative emotions were significantly improved in both the control and intervention groups compared to admission, but the improvement was greater in the experimental group.

### 5.2. Comparison of Satisfaction Rate and Readmission Rate of Two Groups of Chronic Heart Failure Patients Based on IMB Health Education

As can be seen from Figure 7, the satisfaction of health education of heart failure patients in the two groups was compared, and the satisfaction of the intervention group was higher, accounting for about 85.3%, and the dissatisfaction only accounted for 14.3%. The short-term readmission probability was 8.9%. In contrast, the satisfaction of the control group was lower than that of the intervention group, about 67.9%, and the dissatisfaction with health education and the probability of short-term readmission were higher than those of the intervention group, 32.1% and 23.2%, respectively.

The article "Influence of Health Education Based on IMB on Prognosis and Self-Management Behavior of Patients with Chronic Heart Failure" was retracted in 2023. Reasons: unreliable results or conclusions; lack of ethics approval or compliance; concerns about the data; concerns about the peer review.

### 5.3. Comparison of Self-Care Behavior of Two Groups of Patients Based on IMB Health Education

From the self-care situation table in Table 4, the total and maintenance scores of self-care in the intervention group were significantly higher than those before the intervention. The total score and maintenance score of self-care in the control group were also higher than those before the intervention, but the scores of self-care management and self-care confidence were not significantly different, and *P* > 0.05, which was not statistically significant.

Figure 8 shows the comparison of risk perception between the control group and the intervention group before and after the intervention. The results showed that before the intervention, the *P* values of the two groups of heart failure patients in terms of economic risk, physical diagnosis and treatment risk, and psychosocial risk were >0.05, which was not statistically significant. After the intervention, the risk perception *P* value of the two groups of patients was >0.05, which was not statistically significant.

Paired sample *t*-tests were used to compare sentiment scores at baseline, six months, one year, and two years later, as well as data on readmissions between the two groups.

From the data in Figure 9(a), the emotional scores of patients in both groups showed an upward trend with time. But from a detailed point of view, the emotional score of the intervention group was the lowest in the half-year period, only 3.1, and then, although it increased, it was still lower than the baseline level. In contrast, the emotional scores of the control group gradually leveled off after increasing over time. The comparison chart in Figure 9(b) clearly shows the number of readmissions in the two groups. The number of readmissions in both groups also showed an upward trend over time, but the increase in the intervention group was significantly lower than that in the control group.

### 5.4. Interventions to Improve the Quality of Life of Patients with Chronic Heart Failure

1. Psychological intervention: listen carefully to the patient's chief complaint, respect the patient, pay attention to protecting the patient's privacy, put yourself in the shoes of the patient to understand the inner thoughts that cause the patient's negative emotions, give answers and suggestions to the patient, shorten the patient's hospital stay as much as possible, and reduce their economic burden
2. Cognitive intervention: improve patients and their families' awareness of chronic heart failure and correct misconceptions. They should also be made aware of and actively intervene in various risk factors and avoid risky behaviors and predisposing factors to improve disease and quality of life and prevent further disease progression
3. Nutritional intervention: good nutritional self-management can effectively improve patients' compliance with medical treatment, regulate individual behavior, enhance self-confidence, delay the development of disease, and improve quality of life and survival rate
4. Medication intervention: inform patients and their families of the names, doses, uses, effects, and adverse reactions of commonly used drugs to improve their knowledge of medication. Educate them about common adverse effects of the medications they take, and suggest family members to help monitor patients' medication and improve their compliance
5. Exercise intervention: numerous studies have confirmed that proper exercise can improve physical function. The role of exercise rehabilitation in patient rehabilitation and treatment has been widely recognized. It can improve the patient's cardiopulmonary function, improve the patient's exercise tolerance and amount of exercise, and improve the patient's quality of life

The article "Influence of Health Education Based on IMB on Prognosis and Self-Management Behavior of Patients with Chronic Heart Failure" was retracted in 2023. Reasons: unreliable results or conclusions; lack of ethics approval or compliance; concerns about the data; concerns about the peer review.

## 6. Conclusions

The research model of this paper is based on IMB, the experimental samples are divided, and effective health education guidance is provided to the intervention group on the basis of group formation. There are also some innovations in the health education guidance. It has introduced the health education model of cooperation between doctors and nurses from the original nursing care of only nurses. The experimental results show that the health education model can effectively improve the quality of life of patients with chronic heart failure, improve the patient's compliance behavior, improve the negative emotions of patients with chronic heart failure, and promote the recovery of the disease. It can better meet the health education needs of patients, improve the quality of health education, and can effectively improve the satisfaction rate of patients when they are discharged from the hospital, and reduce the readmission rate in a short period of time. It is worthy of clinical promotion and application. From the research data in this paper, the impact on patients with chronic heart failure is mainly reflected in two aspects. First of all, the risk perception of patients is relatively high, and the main factors affecting the risk perception of patients are education, gender, type of expense, and work status. Second, the health education model based on the IMB medical cooperation model can reduce patients' overall risk perception, improve their self-management ability, and deal with disease stress with a more positive attitude. However, the data source for this study was a single site and resided in the same area, which may limit interpretation of the results.

The article "Influence of Health Education Based on IMB on Prognosis and Self-Management Behavior of Patients with Chronic Heart Failure" was retracted in 2023. Reasons: unreliable results or conclusions; lack of ethics approval or compliance; concerns about the data; concerns about the peer review.

## Figures and Tables

**Figure 1:** Schematic diagram of median filtering.

**Figure 2:** Schematic diagram of two-dimensional image gray difference.

**Figure 3:** The basic flow of medical image extraction and classification.

**Figure 4:** IMB mode process.

**Figure 5:** Improved research framework based on the original IMB.

**Figure 6:** Comparison of the symptoms of heart failure between the two groups.

**Figure 7:** Satisfaction of the two groups of patients with health education and the probability of short-term readmission.

**Figure 8:** Comparison of risk perception between control group and intervention group before and after intervention.

**Figure 9:** The emotional changes of the two groups of patients over time and the number of readmissions.

**Table 1:** Basic information of the two groups of patients.

Normal information		Control group	Intervention group	*P*
Gender	Male	31 (55.4%)	26 (46.4%)	0.35
	Female	25 (44.6%)	30 (53.6%)	

Average age		64.3 ± 15.5	64 ± 18.5	0.91

Education level	College degree and above	12 (21.4%)	14 (25%)	0.99
	Middle school or high school	16 (28.6%)	15 (26.8%)	
	Elementary school and below	28 (50%)	27 (48.2%)	

Family monthly income	<2000	19 (33.9%)	16 (28.6%)	0.74
	2000-4000	27 (48.2%)	32 (57.1%)	
	>4000	10 (17.9%)	8 (14.3%)	

Expense reimbursement method	Medical insurance	19 (33.9%)	21 (37.5%)	0.97
	Rural cooperative	22 (39.3%)	22 (39.3%)	
	Poor	8 (14.3%)	7 (12.5%)	
	Own expense	7 (12.5%)	6 (10.7%)	

Profession	Worker	6 (10.7%)	12 (21.4%)	0.29
	Farmer	27 (48.2%)	20 (35.7%)	
	Other	10 (17.9%)	8 (14.3%)	
	Unemployed	7 (12.5%)	12 (21.4%)	
	Retire	6 (10.7%)	4 (7.1%)	

**Table 2:** Comparison of negative emotions between the two groups of patients on admission.

On admission		
Content	Control group	Intervention group
Concern	3.1 ± 0.4	3 ± 0.5
Negative emotions	3 ± 0.5	2.9 ± 0.4
*t*	0.6	1.15
*P*	0.55	0.25

**Table 3:** Comparison of the negative emotions of the two groups of patients at the time of discharge.

On discharge		
Content	Control group	Intervention group
Concern	2 ± 0.5	1.8 ± 0.5
Negative emotions	2 ± 0.4	1.7 ± 0.5
*t*	3.4	3.36
*P*	0.001	0.001

**Table 4:** Comparison of self-care behaviors of two groups of patients with heart failure.

Group	Project	Before intervention	After the intervention	*t*	*P*
Intervention group	Self-care total score	137.5 ± 28	186.4 ± 22	-21.7	<0.001
	Self-care maintenance	46.8 ± 10	60.4 ± 8.6	-14.3	<0.001
	Self-care management	43.8 ± 11.4	64 ± 10.6	-20.68	<0.001
	Self-confidence	47 ± 11	62 ± 9.6	-9.3	<0.001

Control group	Self-care total score	135.3 ± 18.5	138.7 ± 17.3	-3.1	0.004
	Self-care maintenance	45 ± 9.7	48.2 ± 9.2	-8.7	<0.001
	Self-care management	43.5 ± 10.4	44.4 ± 10.1	-1.14	0.26
	Self-confidence	47.2 ± 10.8	46 ± 9.7	1.3	0.2

The article "Influence of Health Education Based on IMB on Prognosis and Self-Management Behavior of Patients with Chronic Heart Failure" was retracted in 2023. Reasons: unreliable results or conclusions; lack of ethics approval or compliance; concerns about the data; concerns about the peer review.

## Data Availability

The data that support the findings of this study are available from the corresponding author upon reasonable request.
